# Overview of Several Typical Ceramic Materials for Restorative Dentistry

**DOI:** 10.1155/2022/8451445

**Published:** 2022-07-18

**Authors:** Hao Yu Shi, Runxuan Pang, Jing Yang, Di Fan, HongXin Cai, Heng Bo Jiang, Jianmin Han, Eui-Seok Lee, Yunhan Sun

**Affiliations:** ^1^Department of Dental Materials, Peking University School and Hospital of Stomatology, National Center of Stomatology, National Clinical Research Center for Oral Diseases, National Engineering Laboratory for Digital and Material Technology of Stomatology, Beijing Key Laboratory of Digital Stomatology, Research Center of Engineering and Technology for Computerized Dentistry Ministry of Health, NMPA Key Laboratory for Dental Materials, Beijing 100081, China; ^2^The Conversationalist Club, School of Stomatology, Shandong First Medical University & Shandong Academy of Medical Sciences, Jinan, Shandong 250117, China; ^3^Department and Research Institute of Dental Biomaterials and Bioengineering, Yonsei University College of Dentistry, Seoul 03722, Republic of Korea; ^4^Department of Oral and Maxillofacial Surgery, Graduate School of Clinical Dentistry, Korea University, Seoul 08308, Republic of Korea

## Abstract

With the development of ceramic technology, prosthodontic ceramics are becoming a useful option for improving esthetic outcomes in dentistry. In this paper, various ceramic materials were reviewed and evaluated, and their advantages and disadvantages and indications in oral prosthodontics were analyzed objectively. The properties of resin-based ceramics, polycrystalline ceramics, and silicate ceramics were compared and analyzed. Resin-based ceramics may replace other ceramic materials in the CAD/CAM field.

## 1. Introduction

With technological advancement of the ceramic field, application of ceramic materials in the field of dental restoration has increased. Ceramic materials have advantages over alloy materials, such as their outstanding optical properties, biocompatibility, low thermal conductivity, color stability, and excellent mechanical properties. Therefore, dental restoration materials have gradually shifted from using alloys to ceramic materials, such as silicate ceramics, polycrystalline ceramics, and resin-based ceramics [1, 2].

Ceramic materials are suitable for subtractive manufacturing, additive manufacturing, hybrid manufacturing (i.e., SM, AM, and HM), and other technologies. Moreover, inlays, veneers, dental implants, all-ceramic crowns, and other restorations made of ceramic materials have been used with long-term clinical success [3].

This paper reviews the literature on ceramic materials and divides the ceramic systems used in the field of dental restoration into three categories: silicate ceramics, polycrystalline ceramics, and resin-based ceramics [4, 5]. Representative ceramic materials in each category are listed and summarized; the classification structure can be seen in Figure 1.

## 2. Silicate Ceramics

Silicate ceramics are nonmetallic inorganic ceramic materials containing a glass phase, which have good optical properties, high transparency, and an attractive and natural appearance. The glass phase and crystal phase of silicate ceramics have different properties. The glass phase is associated with low fracture strength, brittleness, and a nondirectional fracture mode, while the crystal phase can provide advantageous mechanical properties, stability, and esthetics [6, 7].

The most commonly used silicate ceramics in the field of dental prosthetics are feldspar porcelain, leucite-enhanced glass ceramics, and lithium disilicate ceramics. Before bonding silicate ceramics to the tooth structure, the standard ceramic treatment technique is to etch the restoration with hydrofluoric acid, followed by the use of silane coupling agents and dental adhesives [8]. It is worth noting that the concentration of etching agent is not only an important factor affecting the etching strength but also has an effect on the bond strength of the etched material [9]. A study showed that in order to obtain the maximum shear bond strength of silicate ceramics, the concentration of HF acid used for etching is recommended to be 5% or 9% and the etching time should be between 15 and 60 s (etching time and concentration may be adjusted according to ceramic composition and experimental content), but considering that higher concentrations of hydrofluoric acid have higher toxicity, lower concentrations of hydrofluoric acid solutions should be preferred where necessary to meet [9, 10]. Leucite-reinforced ceramics and lithium disilicate ceramics are excellent representatives of high-strength glass ceramics, which have good tolerance to oral environmental conditions such as humidity, pH, and temperature changes [3, 6]. Compared to metal prostheses, ceramic prostheses have lower thermal conductivity and avoid the symptoms of metal allergy in patients. Compared to composite resins, they can reduce the accumulation of plaque and have better biocompatibility with periodontal tissue [1].

### 2.1. Feldspar Porcelain

Feldspar is a common aluminosilicate ore containing calcium, sodium, and potassium. Feldspar porcelain is a kind of traditional ceramic material. It is made of feldspar as the main raw material and sintered with quartz, kaolin, and small amounts of borax and colorants [11].

The main feldspar used in feldspar porcelain is plagioclase, a type of light gray or white crystal, which can be found in rocks abundant in mica and iron [11]. As the raw material for making feldspar porcelain, feldspar must have impurities such as iron and mica removed. When removing impurities, feldspar is crushed and ground, and then, related iron compound impurities are removed using a strong magnet [6, 11]. Kaolin is easy to combine with feldspar. It can be used for the synthesis of dental ceramics to bond ceramic particles together to increase the toughness of the ceramics. However, kaolin is opaque. To ensure the beauty and naturalness of the ceramics, the ratio of kaolin should not be too high [6, 11]. Quartz components can increase the strength of ceramic materials and improve translucency, and borax can act as a solvent. The use of colorants can adjust the color and gloss of the porcelain.

Traditional feldspar porcelain is considered to be the ceramic material with the highest translucency. It has the best optical properties and is the “gold standard” in dental esthetics. Feldspar porcelain is clearly the most suitable type of ceramic for meeting the highest esthetic needs [12, 13]. With the development of minimally invasive technology and the emphasis on restoration esthetics, feldspar porcelain has become an important material for porcelain veneer repair, especially for partial veneers. For example, although zirconia has excellent mechanical properties and high biocompatibility, the all-porcelain crown and the frame made of it for fixing partial dentures usually require feldspar porcelain as the veneer in order to meet the esthetic needs of patients [14].

The service life of feldspar porcelain restorations is considerable. Most of the feldspar porcelain used for inlays can maintain a service life of about 10 years, and most of the integral tooth crowns made of feldspar porcelain or restorations for posterior tooth crowns can maintain a service life of about 12 years [13, 15]. Polishing and glazing can change the roughness of the ceramic surface, reduce the sharpness and pore depth of the restoration surface, and improve the ability of the restoration to resist fracture [16, 17]. A study showed that the fracture load of restorations based on leucite-reinforced glass ceramics was higher than that of ceramic restorations based on feldspar porcelain, but lower than that of all-ceramic restorations based on lithium disilicate glass ceramics, as shown in Table 1 [17].

However, the brittleness and low strength of feldspar porcelain make it more susceptible to damage during clinical operation and processing. For example, when it is used for veneers, it is susceptible to fracture and excessive wear. It is also prone to problems such as fracture restoration and dental crown edge caries when it is used for implants [3, 12, 15, 18]. Due to the reduction in the survival rate of the restoration when it is used in the posterior area of the oral cavity, it is recommended to use feldspar porcelain in the anterior area of the oral cavity [13].

In terms of added ingredients, leucite and fibers were initially used to strengthen feldspar porcelain. In recent years, the use of nanoparticles to improve the strength of feldspar porcelain has been explored. It was found that adding appropriate concentrations of silver and titanium nanoparticles into the feldspar porcelain can improve the strength of the feldspar porcelain and reduce the fracture and notch of the restoration. However, this processing method adversely may affect the color of the feldspar porcelain, and the concentration of nanoparticles should not be too high. High concentrations of silver and titanium nanoparticles will reduce the fracture resistance of the feldspar porcelain [19].

Generally speaking, although feldspar porcelain has shortcomings, it is esthetically pleasing (as shown in Figure 2) and is still widely used in veneers, inlays, crowns, etc. [3].

### 2.2. Leucite-Reinforced Glass Ceramics

Leucite-reinforced glass ceramics are a kind of glass ceramic developed in the 1960s. The addition of leucite crystals increases the crystal content of the ceramic, which helps absorb fracture energy and reduce crack generation and propagation. This improves the strength and fracture toughness of leucite-reinforced glass ceramics while maintaining good semitransparency [6, 7].

The serious mismatch of the thermal expansion coefficients between the frame metal alloy and veneer ceramics in the 1960s promoted the development of leucite and feldspar ceramics. Researchers added leucite into the crystalline phase of feldspar ceramics to improve the mechanical properties [11]. Leucite crystals can be formed by firing feldspar at 1150°C. When the crystal phase is formed, potassium aluminum silicate will decompose into silicon dioxide and leucite [6, 11].

(1) $$\begin{array}{c} {\text{K}}_{2}\text{O}\cdot {\text{Al}}_{2}{\text{O}}_{3}\cdot 6\text{Si}{\text{O}}_{2}⟶{\text{K}}_{2}\text{O}\cdot {\text{Al}}_{2}{\text{O}}_{3}\cdot 4\text{Si}{\text{O}}_{2}+2\text{Si}{\text{O}}_{2} \end{array}$$

Leucite crystals are preferentially etched by acid compared to glass matrix, which makes leucite glass ceramics more likely to form surface characteristics that are easier to be bonded by resin. It makes itself much suitable for making the veneer of metal frames. Thermal residual stress plays an essential function in the mechanical properties of glass ceramics. The mechanical properties of glass ceramics are determined by their composition, microstructure, and type of residual stress (tension or compression) and the magnitude of the residual stress. The effect of thermal residual stress is considered to be the key factor for strengthening leucite glass ceramics. This stress is caused by thermal expansion and the elastic mismatch between the crystal and glass phases after glass ceramics are cooled. The state of residual stress in leucite-reinforced glass ceramics is conducive to improving its strength and toughness [21].

In the field of oral prosthodontics, leucite-reinforced ceramics are widely used in veneer (as shown in Figure 3) and high-strength ceramic prosthodontics [22].

In terms of esthetics, although feldspar porcelain is generally considered to be the most semitransparent ceramic material, there is a research showing that processable leucite-reinforced ceramics have higher semitransparency than processable feldspar porcelain. Leucite-reinforced ceramics also have an excellent esthetic effect. It is suitable for clinical cases with high esthetic requirements. It is also a good material for use in non-load-bearing areas [3, 6, 7].

The service life and success rate of leucite-reinforced glass ceramic dental restoration used in the posterior part of the oral cavity are higher than those of feldspar ceramics. A survey has shown that all-ceramic crowns made of high-strength ceramic materials such as leucite-reinforced glass ceramics and lithium disilicate-enhanced glass ceramics have higher survival rates within five years after oral restoration than those all-ceramic crowns made of feldspar porcelain [14]. Another survey showed that leucite-reinforced glass ceramic crowns had a high survival rate of 79.6% after 13-15 years, indicating that leucite-reinforced glass ceramic crowns can be used as a treatment option for restoring anterior and posterior teeth [24]. In addition, inlay and onlay restorations made of leucite-reinforced glass ceramic have shown satisfactory clinical results with a failure rate of about 16% after 12 years and no secondary caries observed [25]. However, due to the nature and machinability of leucite-reinforced glass ceramic, some studies still do not recommend its use in posterior dental crowns and fixed dentures [7, 26, 27]. There are various factors that affect the life of ceramic restorations. The constant change of saliva pH, acidic beverage, and dental plaque can increase the surface roughness, damage the glaze layer, and reduce the ceramic thickness, thus reducing the fracture strength and fracture toughness of the ceramics. Additionally, roughening of restorations also increases wear on tooth enamel and increases the incidence of oral diseases, such as chronic gingivitis caused by plaque buildup [28, 29]. It is worth mentioning that when the patient has the need to reduce the cost and time of treatment or the desire to extend the life, appearance, and function of the original implant, the patient's needs can be met by bonding the new restoration to the original restoration with an adhesive [30]. This method is low cost and efficient and not only improves the restoration beyond esthetics and function but also effectively improves the problem regarding the high rate of veneer ceramic breakage [30].

Surface treatment technology can improve the properties of leucite-reinforced glass ceramic restorations. The bending strength of leucite-reinforced ceramics can be improved by glazing, and the surface smoothness of leucite-reinforced ceramics can be improved by polishing. Both techniques can reduce the occurrence rate of crack or the depth of crack on ceramic surface [11, 28].

Benefiting from the high biocompatibility, high flexural strength, and esthetics of leucite-reinforced glass ceramics, such ceramics are widely used in the field of prosthodontics [11, 28].

### 2.3. Lithium Disilicate Ceramics

Lithium disilicate ceramics are composed of lithium disilicate crystals and a glass matrix. The crystal phase content of ceramics accounts for the majority of the total ceramic and the glass phase content is relatively small, which makes it excellent mechanical properties and fracture toughness. It also has a high esthetic and good bonding strength and is one of the most widely used nonmetallic materials [8, 11].

When producing lithium disilicate, the ceramic is first cast in a transparent glass ingot containing lithium orthosilicate (Li_4_SiO_4_), and then, the crystalline lithium metasilicate crystal (Li_2_SiO_3_) is embedded in the glass phase. At this time, the formed block is easy to mill and has a bending strength of 130 ± 30 MPa. The milled restorations are then tempered at 850°C to form lithium disilicate crystals (Li_2_Si_2_O_5_). The bending strength of lithium disilicate ceramics can reach 360 ± 60 MPa, and dense lithium disilicate crystals can be seen after hydrofluoric acid is used to dissolve the glass matrix on the surface (the image of lithium disilicate ceramics etched by hydrofluoric acid is shown in Figure 4) [6]. A comparison of other relevant properties is shown in Table 2.

One of the advantages of lithium disilicate ceramics is that lithium disilicate ceramics can be reduced to a certain thickness while still maintaining high strength (ceramic thickness, restoration geometry, and bonding technology are the key factors affecting ceramic properties, and the opacity and thickness are directly related [1, 32]), enabling it to maintain excellent mechanical properties and esthetics at a specific thickness. And it can look natural by tinting (as shown in Figure 5). The excellent biomechanical properties make it suitable for posterior crown, all-porcelain bridges, and short-span fixed partial dentures. Multiple experiments, clinical trials, and laboratory reports have shown that lithium disilicate ceramics have good restorative effects [3, 11].

Although lithium disilicate ceramics are less attractive in their appearance than feldspar porcelain, they are often used to construct the core of restorations and are an important substitute for metal due to their higher bending strength and fracture toughness. The color stability of lithium disilicate ceramics can be improved through glazing procedures. Additionally, in cases where the use of feldspar porcelain materials in the posterior area of the mouth is not recommended, lithium disilicate ceramics have shown excellent and long-term success in the anterior region and posterior region of the oral cavity, such as extended veneers (as shown in Figure 6) [33]. Therefore, the excellent mechanical properties, high flexural strength, and esthetic properties of lithium disilicate ceramics make it the first choice for the overall restoration of the posterior oral area and gradually become one of the most popular all-ceramic restoration materials [7, 11, 13, 26].

On the whole, the prospects of silicate ceramics are still bright, with many advantages such as stable color, low thermal conductivity, good wear resistance, and high biocompatibility. These materials remain indispensable in oral restoration. They are used in decorative alloys, single tooth prostheses, full contour crowns, and other aspects. They are also suitable for SM and AM, although the AM process is more complicated, which may cause cracks due to cooling and increase the porosity of the ceramic interior and reduce the mechanical properties. Hybrid manufacturing (HM), utilizing a combination of CAD/CAM and 3D printing, will be an interesting endeavor to make dental restorations [3, 18, 22, 27].

## 3. Polycrystalline Ceramics

Polycrystalline ceramics are manufactured by sintering, and they are also generally referred to as sintered ceramics.

Among chairside digital prosthetic materials, polycrystalline ceramics are generally stronger mechanically than glass ceramics. They are a popular class of materials used in chairside digital prosthetics today. In polycrystalline ceramics, no glass phase is present and all crystals are arranged in a dense conventional matrix. This arrangement limits the extension of cracks and provides them with superior mechanical properties [35]. Additionally, the absence of a glass matrix allows the ceramics to possess resistance to surface etching with hydrofluoric acid [36]. Polycrystalline ceramics, which usually have low transparency due to the lack of a glass phase, are mostly used for the manufacture of crowns and bridges, which are then fitted with veneering porcelain to improve the esthetics [37]. Currently, polycrystalline ceramics that are frequently employed in dental restorative materials include alumina ceramics and zirconia ceramics.

### 3.1. Alumina Ceramics

Alumina ceramics are ceramic materials in which aluminum oxide (Al_2_O_3_) is the main component. By chemically treating bauxite, raw alumina can be obtained with extremely high purity.

The main crystalline phase of alumina ceramics is corundum (AI_2_O_3_), which has four isomorphs: *α*-Al_2_O_3_, *β*-Al_2_O_3_, *γ*-Al_2_O_3_, and *δ*-Al_2_O_3_. The *α*-Al_2_O_3_ crystalline form has the best thermal and chemical stability [38]. This is essentially the only form of alumina that is currently used in the field of dental prosthetics. Depending on the content of alumina in alumina ceramics, they can be classified into two categories: high-purity type and normal type. Ultrapure alumina ceramics contain more than 99.9% alumina and have excellent characteristics such as porosity, high dispersion, insulation, and heat resistance [39]. Ordinary alumina ceramics are divided into different varieties according to their alumina content, such as 99 porcelains, 95 porcelains, 90 porcelains, and 85 porcelains. In some cases, ceramics with a content of approximately 80% or 75% alumina are also classified as ordinary alumina ceramics. In alumina ceramics, the mechanical strength decreases as the content of alumina decreases. Thermal conductivity also increases with increasing alumina content. The alumina content of alumina ceramics used in dental restorative materials is generally above 50 wt%, where the alumina ceramics have good mechanical strength and their bending strength increases with increasing alumina content [40].

Regarding the sintering of alumina ceramics, this process is usually performed using ultrafine powders with good sintering activity and adding appropriate amounts of sintering aids to lower the sintering temperature required to obtain ceramics with excellent mechanical properties. The usual sintering aid added to alumina ceramics is MgO, which effectively inhibits excessive grain growth and tends to make the sintering completely dense. For ceramic materials, the sintering temperature can generally be reduced by using both ultrafine powders and sintering aids, and the reduction in the sintering temperature results in a ceramic material with excellent mechanical properties [41].

Alumina ceramics have a very high hardness and density, and their Mohs hardness reaches nine, which is slightly lower than diamond. In medicine, they are often used to make dental prosthetic materials and artificial joints (e.g., hip joint balls). Studies have shown that the Rockwell hardness of alumina ceramics is approximately HRA80-90, while the bending strength of sintered and hot-pressed products can reach 250 MPa and 500 MPa, respectively [42].

As the standard of living around the world improves, more and more people are paying attention to the esthetics of their teeth. Thus, we normally try to ensure attractive esthetics in the restoration of teeth. Because of their similar color and natural luster to real teeth, alumina ceramics are commonly used to make crowns, bridges, and veneers for anterior teeth. The use of alumina all-ceramic crowns can achieve better cosmetic restorative dentistry than zirconia all-ceramic crowns and effectively reduce the likelihood of gingivitis. However, alumina ceramics have a high modulus of elasticity, reaching 380 GPa, which makes them prone to fracture [43]. There is currently no complete solution to this problem, which is one of the reasons for the gradual replacement of alumina ceramics by zirconia ceramics. The use of zirconia is significantly more effective than the use of aluminum oxide for the restoration of posterior areas of the oral cavity.

Aluminum oxide is currently a widely used restorative material in clinical practice. Choosing the bonding agent is very important for all-porcelain alumina crowns. The bond strength can directly affect the restorative effect of an all-ceramic crown, and the use of different bonding agents will produce different bond strengths [44]. Currently, commonly used bonding agents for alumina crowns include the Fuji multipurpose glass ionomer and flowable composite resins. In contrast, the bonding of alumina crowns can be made stronger with flowable compound resin bonding agents; these have a higher clinical application value.

The first completely intensive dental polycrystalline ceramic was Procera™ AllCeram (Nobel Biocare, Göteborg, Sweden), introduced in 1993. Procera™ AllCeram has a transparency between Empress™ 1 and Empress™ 2 and has been tested to have a consistent marginal fit of 60-80 *μ*m, which is within the clinically acceptable range [45]. In a six-year evaluation of the clinical use of Procera™ AllCeram single crowns, the accumulated survival and success rates over six years were 95.2% and 90.9%, respectively, which is a great advantage for clinical use [46].  Figure 7 shows the patient's recovered portion of the broken Procera™ AllCeram premolar crown and the SEM image of the Procera™ AllCeram. In-Ceram AL appeared, made by VITA Zahnfabrik, also a representative example of an alumina ceramic. It has a higher mean fracture load [941.8 (±221.66) N] (*p* > 0.05) compared to other ceramic materials like IPS-Empress II and Top-Ceram (a more detailed comparison of some of the properties of the three materials is shown in Table 3) [47]. In-Ceram alumina is a suitable material for anterior and posterior crowns, as well as for anterior single-retainer RBFPD. Certain other specific data for the two alumina ceramic products are shown in Table 4.

Normally, the microstructure of alumina ceramics consists of isometric particles, with a polycrystalline structure consisting of ionic or covalent bonds. Therefore, the fracture toughness of alumina ceramics is low. Under the action of external forces, the stress will cause fine cracks on the surface of the ceramic, and the rapid expansion of cracks makes alumina ceramics undergo brittle fracture. Toughening research is a central topic in the study of alumina ceramic materials. Currently, there are a few main methods used to improve the fracture toughness of alumina ceramics: particle dispersion toughening, fiber and whisker toughening, zirconia phase change toughening, composite toughening, and self-toughening. Today, alumina ceramics are often toughened by zirconia phase change toughening, and ceramics toughened by this method are called zirconia-toughened alumina ceramics (ZTA). The process involves adding Y-TZP (yttrium-oxide-stabilized zirconium oxide) to the alumina matrix and distributing it evenly throughout the alumina matrix to achieve a good toughening effect. A study of the wear and corrosion phenomena on the toughened alumina ceramics showed that the wear and corrosion resistance of ZTA was superior to that of yttrium-oxide-stabilized zirconium oxide (YSZ) [51]. The clinical application of ZTA has also been investigated, with Larsson et al. [52] conducting a five-year follow-up study of implantable ZTA (using the In-Ceram Zirconia, VITA Zahnfabrik [InZ] repair system), which showed considerable clinical advantages. The In-Ceram Zirconia repair system is illustrated in Figure 8.

In recent years, due to the advent of zirconia ceramics and their superior physical and chemical properties, alumina ceramics have been gradually replaced by zirconia ceramics in the field of restorative dentistry. However, compared to zirconia ceramics, alumina ceramics still have advantageous characteristics, in that they are very stable at high temperatures and in physiological fluids. In conclusion, alumina ceramics may still have a promising future in the field of prosthodontics.

### 3.2. Zirconia Ceramics

In the early 1990s, zirconium oxide was introduced into the field of denture processing, and today, it is a popular material in the field of dentistry. In general, zirconia is yellow or gray in color, although high-purity zirconia is white.

Today, zirconia ceramics are a popular type of dental restorative ceramic on the market. At atmospheric pressure, pure zirconia has three crystalline forms: monoclinic zirconia (m-ZrO_2_), tetragonal zirconia (t-ZrO_2_), and cubic zirconia (c-ZrO_2_).  Figure 9 shows transmission electron microscopy images and high-resolution transmission electron microscopy images of the three crystal forms. The material changes forms at different temperatures. At temperatures less than 1170°C, zirconia is in the monoclinic (m) phase with a density of 5.65 g/cc. The tetragonal (t) phase occurs from 1170°C to 2370°C with a density of 6.10 g/cc, and the cubic (c) phase occurs above 2370°C with a maximum density of 6.27 g/cc [53, 54]. Zirconia is most stable when it is in the monoclinic (m) phase. Under certain conditions, zirconia undergoes the t-m transition. When this transition occurs, the volume of zirconia also changes. This change is known as “tensorial expansion,” which is a phenomenon that occurs widely in steel. Hence, zirconia is also known as “ceramic steel” [55]. During the t-m transformation process, zirconia's stability can be enhanced by limiting crack extension through the expansion of the particle volume, which is limited by the surrounding material. This phenomenon is known as “stage transformation strengthening.” The flexural strength of partially stabilized zirconia is generally in the range of 1600-2100 MPa and a modulus of elasticity of approximately 200-210 MPa [56]. Zirconia ceramics have a very high mechanical strength at normal temperatures. As a result of the excellent properties of zirconia ceramics, they are currently used in clinical practice for prefabricated root canal crowns, single crowns, all-ceramic crowns, and all-ceramic crown and bridge restorations.

As a biologically inert ceramic, the biocompatibility of zirconia ceramics is clearly excellent, enabling the emergence of zirconia implant abutments. In 2006, zirconia implant abutments were officially used in clinical practice for the first time. Compared to metallic materials, zirconia implant abutments offer better esthetic results and can restore the color of natural teeth to a greater extent. Additionally, the lower surface free energy and wettability of zirconia abutments can effectively reduce the risk of periodontal inflammation after implantation [58].

Although the mechanical properties of zirconia are quite good, the optical properties are relatively poor. The installation of veneered porcelain is usually required to achieve an adequate esthetic effect, and using micromechanical inlays is the main method of bonding between veneer porcelain and zirconia. Although the use of veneers satisfies the desired esthetic effect, veneers are prone to chipping. Currently, a major cause of clinical failure of zirconia restorations is disintegration of the veneer [59].

For the treatment of zirconia ceramic surfaces, alumina blasting techniques are often used in clinical settings to treat the ceramic surface. However, for zirconia, the alumina blasting technique does not dramatically improve the bond strength on the zirconia surface. It has been demonstrated that sandblasting causes microcracks on the surface of the zirconia material, reducing the mechanical properties of the zirconia material itself [60]. As a result, the alumina blasting technique may not be the best option for zirconia. Some experiments have shown that silicon nitride blasting may be more effective than alumina blasting for zirconia, and further investigation is required to compare the effects of these two types of blasting [61].

For the processing of zirconia ceramics, zirconia is currently processed by CAD/CAM systems, such as CEREC, PROCERA, and KAVO (Figure 10 illustrates the basic flow of a CAD/CAM system) [62]. These systems first use zirconia powder to form the molded body. This is followed by sintering at a lower temperature to obtain a zirconia presintered body, cutting the presintered body to obtain a presintered zirconia inner crown, and finally sintering at a higher sintering temperature to precisely control its shrinkage to obtain a dense zirconia denture. This method has greatly improved the processing efficiency of zirconia prostheses and has led to the promotion of zirconia as a dental prosthetic material.

In order to obtain different types of zirconia ceramics, we usually need to add different types of stabilizers, such as CaO, MgO, Y_2_O_3_, and CeO_2_. The most widely used stabilizer is Y_2_O_3_. In 1976, researchers first observed that t-ZrO_2_ could be made stable or substable at room temperature by adding Y_2_O_3_. Later, it was experimentally demonstrated that TZP ceramics with a fully tetragonal phase could be formed by stabilizing zirconia with 2 mol% to 3 mol% Y_2_O_3_ [64].

Commercially applied zirconia is mostly found in various products as tetragonal zirconia polycrystals (Y-TZP), which must be polished after grinding to ensure adequate mechanical properties in the Y-TZP ceramics [65]. Y-TZP can be broadly divided into two types of material depending on the process technique: hot isostatic compression (HIP) and cold isostatic compression (CIP). More zirconia powder is required to use HIP than CIP, but the strength of zirconia ceramics made using the HIP process is 20% stronger than those made using the CIP process. Procera uses HIP-type zirconia.

One of the biggest drawbacks of zirconia ceramics is their low-temperature ageing. Kobayashi et al. [66] first suggested that Y-TZP undergo a slow t-m phase transition at 250°C in a moist environment, which is essentially a martensitic phase transition followed by a significant reduction in the mechanical properties. The primary elements impacting zirconia aging are the type and amount of stabilizer added inside the zirconia ceramic, the grain size, and the residual stress.

Many discussions have been made about the mechanism of low-temperature ageing. Currently, one of the widely accepted ageing mechanisms is the point defect reaction ageing mechanism based on oxygen vacancies and water molecules [67]. This ageing mechanism can be represented by the following two chemical equations.

(2) $$\begin{array}{c} {\text{H}}_{2}{\text{O}}_{\text{ad}}+{\text{O}}_{\text{surf}}^{2-}⟶2\text{O}{\text{H}}_{\text{surf}}^{-} \end{array}$$

(3) $$\begin{array}{c} 2\text{O}{\text{H}}_{\text{surf}}^{-}+\text{V}\ddot{\text{o}}⟶{\left(\text{OH}\right)}_{\text{o}}+{\text{S}}_{0\text{surf}}^{\text{X}} \end{array}$$

Reaction (2) describes the process of breaking the space structure bonds of zirconia, while reaction (3) describes the process by which hydroxyl groups move and diffuse on the surface of zirconia, thereby forming defects.

It has been found that Y-TZP has excellent ageing resistance when the zirconia grain size is controlled to be 0.3-0.4 *μ*m [68], but the ageing resistance can also be increased by adding various oxides or nonoxides. 3Y-TZP has the best ageing resistance when AI_2_O_3_ is added to it at 0.25 wt% [69]. Alumina-toughened zirconia (ATZ) is a zirconia ceramic composite material formed by adding alumina (*α*-Al_2_O_3_) to zirconia as a matrix. The *α*-Al_2_O_3_ dispersive phase particles contained in the composite can, to a certain extent, hinder the t-m phase transition of 3Y-TZP [70]. The physical and chemical characteristics of ATZ support its application in dental applications, and its resistance to ageing is better than that of 3Y-TZP. However, further research is still required to enhance the hydrothermal stability of ATZ. Kohal et al. [71] evaluated the clinical use of ATZ and found that the survival rate of ATZ implants was 94.3% after five years and that the material had an advantage in terms of bone tissue stability with a bone loss of 0.81 mm over five years. Based on these results, ATZ can be recommended for clinical use.

Fully anatomic zirconia is a hot topic of research in recent years. Fully desorbed zirconia refers to a restoration with a fully desorbed morphology that is designed and manufactured directly from zirconia by CAD/CAM technology. This process eliminates the need for veneering porcelain and reduces the possibility of restoration failure. Fully desquamated zirconia is extremely strong mechanically and does not cause excessive wear on natural teeth because it is less abrasive than feldspathic ceramics [72]. As this technology has evolved, fully destructive zirconia, which was earlier used mainly in the posterior region, has gradually been applied for the esthetic restoration of anterior teeth.

Graded zirconia was also created as a new material in response to the chipping of veneered porcelain. Graded zirconia materials are manufactured by infiltrating glass into 3Y-TZP while sintering it. Due to the penetration of the glass, the graded zirconia ceramics have a better esthetic effect. A study of the wear properties of the new graded zirconia material showed that polished graded zirconia has better wear properties compared to zirconia. It can be inferred that it has adequate clinical wear properties and has a smooth wear surface that can be used to reduce wear on the tooth [73].

VITA In-Ceram® YZ (VITA Zahnfabrik) and Lava™ Frame Zirconia (3M ESPE) are two of the better-known products in the world today. Certain other specific data for the two zirconia ceramic products are shown in Table 4. Both of these materials can be used to make zirconia bridges. Models of the zirconia bridge and the fixed zirconia bridge are shown in Figure 11.

It is undeniable that zirconia ceramics offer excellent physicochemical features compared to many other dental restorative materials (some of the important properties of zirconia and alumina products are compared in Table 4). Although low-temperature ageing of zirconia ceramics due to t-m phase changes in humid, low-temperature environments (or oral environments) can occur, numerous researchers have addressed the issue of low-temperature ageing of zirconia ceramics in various ways. As their resistance to ageing increases, zirconia ceramics are bound to become more widely used in dentistry.

## 4. Resin-Matrix Ceramics

In recent years, with the increasingly mature processing technology of resin-based ceramics and the continuous improvement of their performance, the application of these ceramics in the field of oral prosthodontics has become more and more extensive [77]. Resin-matrix ceramics are a new type of ceramic material that combine the advantages of ceramic and polymer materials. This composite material features a resin matrix based on inorganic ceramics [78].

Resin-based ceramics are a new kind of composite material, although they are not technically ceramics. However, they have similar properties with ceramic materials, including similar esthetics, strength, adhesion, wear resistance, and other characteristics that are very close to those of porcelain.

The composition of resin-based ceramics is more than half inorganic compounds. However, according to the current definition of the International Nomenclature Committee, only “inorganic refractory material as the main body through cutting, sintering, die casting materials can be called ‘porcelain'.” Therefore, resin-based ceramics are not ceramics in the strict sense, but they are ceramic-like materials. And these materials still tend to be called resin-based ceramics [79]. Resin-based ceramics have both ceramic and resin characteristics, and their elastic modulus is low, similar to dentin. Since resin-based ceramics have an elastic modulus comparable to that of dentin, they can be more readily ground and embed in the oral cavity compared to other ceramic materials.

The biggest advantage of resin-matrix ceramics is that they provide fantastic retention force for the side wall and have good stability when used as the crown repair body, inlays, and onlays.

### 4.1. VITA ENAMIC Ceramic (PICN)

In the past few years, CAD-CAM has been used more and more widely in oral cavity applications, whether it is scanning the dentition model of the patient, designing the prostheses needed by the patient, or printing the designed prostheses directly by a printer. Achieved in the field of dental restorations all applications. This is also in line with the high efficiency and digital trend of today's society.

However, during the printing process of the original ceramic materials for oral prosthesis, it is easy to break the material due to its high hardness. Additionally, due to the difficult nature of printing, it is easy to create a prosthesis that does not fit perfectly.

In recent years, VITA has produced a new type of ceramic for oral repair, which solves this problem [5]. The new material is a polymer-permeable ceramic mesh developed based on glass-permeable ceramic technology. The mesh manufacturing process is simple. First, the powder is pressed into small pieces and then fired to form a network of porous ceramics. Next, the ceramic matrix structure is tuned with a coupling agent. The regulated network of the porous ceramic is eventually permeated by the monomer mixture and then thermally induced polymerization forms the polymer network. Both networks are connected to each other through chemical bonds obtained by coupling agents [6]. A representative image of the ENAMIC microstructure is shown in Figure 12.

PICNs have the advantage of having about a 50% lower elastic modulus than feldspar ceramics (closer to dentin). Therefore, they are easier to mill and easier to use when repairing composite resins. The new material has a lower modulus of elasticity and higher resistance to damage than traditional dental ceramics [80].

The composition analysis of the main ceramic network shows that the main ceramic phases consist of SiO_2_ (58-63%), Al_2_O_3_ (20-23%), Na_2_O (9-11%), K_2_O (4-6%), B_2_O_3_ (0.5-2%), CaO (<1%), and TiO_2_ (<1%) [81]. PICN has positive properties in both ceramics and composites. The composite has an interesting balance between flexibility and intensity, making it suitable for individual crowns, inlays, high inlays, and veneers.

As is expected in composites, the properties fall somewhere between the ceramic and particle-filled resin. Compared with traditional veneer ceramics, the elastic moduli of materials that constitute PICN are in the range of 30 GPa, which is closer to common dentin (within the 30 GPa range) [82]. Compared with other CAD/CAM and stamping materials, PICN has a high degree of resistance to grinding damage on diamond drill bits. It has a higher damage tolerance than other ceramics, such as veneer ceramics used in CAD/CAM [83].

Clinical simulation shows that PICN is of great practical value in antifatigue applications. Five years of chewing simulation results showed that all-ceramic crowns made from ENAMIC did not crack. ENAMIC behaves just like lithium disilicate glass ceramics over 500,000 fatigue tests [5]. Due to the reduced modulus of elasticity of ENAMIC, this material is particularly suitable to be used for prosthetic treatment of hard implants. Due to its poor optical characteristics, PICN is more suitable for use in the molar region compared with the anterior tooth region [84].

Dental wear also results in damage to hard tissues from causes other than caries or trauma, and it is a normal physiological process throughout a person's life. Rapid wear of teeth can lead to problems such as dentin hypersensitivity, pulp exposure, and even periapical disease [85]. In many cases, enamel is restored by ceramic or composite materials due to tooth decay, fracture, or external trauma. The material of the prosthesis has a decisive influence on tooth wear [86].

Previous studies have shown that traditional ceramics may cause excessive wear on teeth, resulting in damage to tooth anatomy and morphology, abnormal occlusion curves, and even temporomandibular joint disorder. ENAMIC, as a new type of ceramic material for oral repair, addresses the problems of poor wear resistance, poor aging sensitivity, small leakage, and long-term stability of composite materials. Mechanical properties show that ENAMIC is a better repair material than glass ceramics or resin composites.

Nevertheless, the desired restorative material should have excellent mechanical properties, as well as a wear rate similar to that of tooth enamel [87].

Enamel is more wear-resistant than tooth enamel. The wear pattern of ENAMIC is similar to that of tooth enamel. The polymer phase wears preferentially, similar to the interrod area in enamel rods, and then, the ceramic phase is removed from the wear surface, similar to what happens in enamel rods. Although its wear resistance is lower than that of tooth enamel, it is still superior to other many materials [5].

### 4.2. Resin Nanoceramic

The development of intraoral scanning, quicker and more powerful milling machines, and stronger CAD/CAM materials has led to the innovation and development of indirect prosthetics. As a result, CAD/CAM technology is becoming more common [89]. But it has also created a need for new materials to fill gaps in chairside manufacturing.

Therefore, resin nanoceramics came into being. The material is a mixture of resin and composite materials, which has the advantages of both, but is mainly composed of ceramics. Not only is it not brittle and fracture resistant like composite materials, it also has the advantages of glass ceramics, including excellent gloss retention and long-lasting beauty [6]. This new material is cured at high temperatures through a proprietary, controllable manufacturing process, which eliminates the postmilling baking step. What is more, resin nanoceramics can be easily machined on the edge of a chair or in a dental lab. They can also be quickly polished to an esthetically pleasing surface and can be further adjusted with a photocurable restorative if required.

3M ESPE's Lava Ultimate is recognized as a commonly used resin-based nanoceramic (RNC), which consists of nanoceramic particles combined at a high level in a cross-linked polymer matrix [90].

Lava Ultimate contains two monodispersed and nonaggregate nanopolymers: a 20 nm diameter silica nanopolymer and a 4-11 nm diameter zirconia nanopolymer, which synthesize nanoclusters composed of 20 nm silica and 4-11 nm zirconia. The average particle size was 0.6-10.0 *μ*m. Nano-sized particles allow a high proportion of ceramic fillers (accounting for about 80% of the weight) to be incorporated into the resin [6]. The nanopolymers and nanoclusters are processed using silane coupling agents to form chemical bonds between the ceramic particles and the resin matrix. This material undergoes a special heat treatment process for several hours, resulting in a highly solidified material that does not require further milling after roasting [91].

This procedure is faster than procedures using other CAD/CAM materials because it requires no firing, and it allows for grinding, polishing, and adjustment for improved durability and shock absorption characteristics [90]. Compared with composite materials (nanoclusters), the specific composition and production technology enable these nanoceramics to have a higher bending strength (200 MPa) than CAD/CAM feldspar ceramics and simple composite resins.

It also has better fracture performance and wear resistance, and it significantly improves polishability and optical properties [82]. In the polymer, the resin serves as a matrix to help improve some of the properties of the composite material. For example, the material is not brittle, it is resistant to fracture, and it has characteristics such as shock absorption. However, although the ceramic content is high, this material is not advised for crowns, but only for inlays, high inlays, and veneers. When it is used as a crown, the restoration is prone to break off.

### 4.3. Flexible Nanoceramic

Flexible nanoceramics are a ceramic-like resin material with a nanofiller, as introduced by GC Company of Japan. They have with a flexural strength of 231 MPa [92]. This ceramic is made up of small and uniformly distributed aluminum-barium silicate particles embedded in a polymer matrix. This specific design of the ceramic nanomatrix makes it ideal for high-strength and absorbent restorations for all indications, especially for implant-supported crowns. Figures 13 and 14 are a representative sample of the macrophotographs of the milled crown margins for a resin-based material and its corresponding micrograph.

Due to its dynamic, proprietary nanoceramic matrix and complete homogeneity, CERASMART is a truly self-polishing material. It not only stays polished longer but also is proven to retain its luster even after wear and tear [92]. Compared with other materials, CERASMART can protect the dental post more easily due to its better stress dispersion. This material exhibits an opalescence effect and fluorescence effect that are very close to natural tooth tissue. Before bonding, CERASMART can be sandblasted with alumina (particle size: 25-50 *μ*m, pressure: 0.2 MPa). If there is no sandblasting, it can also be etched with 5% hydronitacid for 60 s and then coated with a silicon coupling agent to enhance the bonding strength [93].

Indications for this material include veneers, inlays, high inlays, single crowns, implant superstructures, and other repair forms.  Figure 15 shows the postoperative intraoral views of the completed composite resin restoration on tooth 9 and chairside CAD/CAM-fabricated crown 8.

With the continued development of resin-based ceramics technology, we believe that resin-based ceramics like this product will become increasingly popular in the field of oral repair in the near future due to the various excellent properties.

## 5. Conclusion

Ceramic materials have become a mainstream material in restorative dentistry. Owing to their outstanding chemical and mechanical characteristics, these can be used in a wide range of clinical situations. The esthetic characteristics of ceramic materials are superior to those of other dental restorative materials.

With the increasing needs of people, ceramic materials have been continuously developed. In addition to traditional silicate ceramics and popular polycrystalline ceramics of recent years, resin-based ceramics are becoming more widely used in dental prosthetics. Silicate ceramics are impeccable in terms of their esthetics, but they are obviously weaker than polycrystalline ceramics and resin-based ceramics in terms of the mechanical properties, so they are currently used to make veneer ceramics. Resin-based ceramics are easier to grind and adjust in the oral cavity than other ceramics due to their elastic modulus (relative to dentin). Polycrystalline ceramics are less translucent, but their mechanical properties are superior, and their esthetic properties compare favorably with other nonceramic restorative materials.

Although ceramic materials can now handle a variety of clinical situations, research into ceramic materials has not stopped, and researchers continue to look for ways to further refine the various characteristics of ceramic materials to better meet the needs of patients. It should be noted that all-ceramic prostheses are not recommended when the patient has poor oral hygiene or periodontal disease. Based on our review of ceramic materials and their current state of development, the future of ceramic materials is bright.

## Figures and Tables

**Figure 1:** Classification of ceramic types in this paper.

**Figure 2:** (a) A feldspar porcelain veneer placed on the model frame [20] and (b, c) feldspar porcelain after sintering and glazing [14].

**Figure 3:** Porcelain veneer of leucite-reinforced glass ceramics [23].

**Figure 4:** Three lithium silicate/disilicate hot-pressed glass ceramics: IPS e.max Press, Initial LiSi Press, and Celtra Press. (a) Etched ingot specimens (IPS e.max Press). (b) Etched ingot specimens (Initial LiSi Press). (c) Etched ingot specimens (Celtra Press) [31].

**Figure 5:** (a) Labial view of lithium disilicate ceramic veneers and (b) palatal view of lithium disilicate ceramic veneers [33].

**Figure 6:** (a) A crystal fired lithium disilicate ceramic crown and (b) the tinted lithium disilicate ceramic crown based on a shaded representation of the patient's other teeth. Both images show the same ceramic crown [34].

**Figure 7:** (a) Recovered part by the patient of a broken Procera™ AllCeram premolar crown. (b) SEM micrograph of the Procera™ AllCeram microstructure after Vickers hardness measurements [48, 49].

**Figure 8:** (a) Radiographic image, (b) frame, and (c) In-Ceram Zirconia (InZ) [52].

**Figure 9:** Transmission electron microscope images: (a) m-ZrO_2_, (b) t-ZrO_2_, and (c) c-ZrO_2_. High-resolution transmission electron microscopy images: (d) m-ZrO_2_, (e) t-ZrO_2_, and (f) c-ZrO_2_ [57].

**Figure 10:** Dental CAD/CAM system process diagram [63].

**Figure 11:** (a, b) Illustrations of a zirconia bridge and a fixed zirconia bridge [74].

**Figure 12:** Micrographs of the ENAMIC microstructure. “C” designates the ceramic phase (light gray) and “P” designates the polymer phase (dark gray) [88].

**Figure 13:** A macroscopic photograph of the buccal margin of the CES restoration. The dashed box indicates the area observed under a light microscope [92].

**Figure 14:** CES repair under optical microscope (50x), showing the buccal margin [92].

**Figure 15:** (a, b) Details of resin-based ceramic restorations [94].

**Table 1:** Comparison of fracture load values between polished and overglazed ceramic plates of several ceramic materials.

Material	Ceramic type (chemical components)	Fracture load values (*N*; mean ± SD)	
		Polished ceramic plates	Overglazed ceramic plates
Vita Mark II	Fine particle feldspar ceramic (SiO_2_, Al_2_O_3_, Na_2_O, K_2_O, CaO, TiO_2_)	591.3 ± 114.9	684.2 ± 152.5
ProCAD	Leucite-reinforced glass ceramic (SiO_2_, BaO, Al_2_O_3_, CaO, CeO_2_, Na_2_O, K_2_O, B_2_O_3_, TiO_2_)	820.2 ± 210.2	818.1 ± 160.6
IPS Empress CAD	Leucite-reinforced glass ceramic (SiO_2_, BaO, Al_2_O_3_, CaO, CeO_2_, Na_2_O, K_2_O, B_2_O_3_, TiO_2_)	858.1 ± 121.9	892.8 ± 123.1
IPS e.max CAD	Lithium disilicate glass ceramic (SiO_2_, Li_2_O, K_2_O, P_2_O_5_, ZrO_2_, ZnO, Al_2_O_3_, MgO)	1,107.9 ± 220.8	1,200.5 ± 304.0

**Table 2:** Partial properties and indications of feldspar porcelain, leucite ceramics, and lithium disilicate ceramics [1, 6, 26].

Ceramic type	Flexural strength (MPa)	Modulus of elasticity (GPa)	Brittleness index (*μ*m^-1/2^)	Vickers hardness (GPa)	Fracture toughness (MPa m^1/2^)	Clinical indications
Feldspar porcelain	154	45	2.31 ± 0.11	5.97 ± 0.22	1.39 ± 0.23	Veneers, inlays, onlays, partial crowns, anterior and posterior crowns, CAD/CAM materials
Leucite ceramics	160	62	1.77 ± 0.11	5.74 ± 0.20	1.43 ± 0.26	Veneers, onlays, inlays, partial crowns, anterior and posterior crowns, CAD/CAM materials
Lithium disilicate ceramics	360 ± 40	95	2.53 ± 0.17	6.84 ± 0.16	2.18 ± 0.23	Veneers, inlays, onlays, partial crowns, anterior and posterior crowns, CAD/CAM materials, three-unit bridges (anterior and premolar), hybrid abutments, hybrid abutment crowns

**Table 3:** Comparison of some properties of the three materials [50].

	In-Ceram alumina	IPS-Empress II	Top-Ceram
Manufacturer	Vident, Brea, CA, USA	Ivoclar Vivadent, Amherst, NY, USA	Global Top Inc., Goyang-si, Gyeonggi-do, Korea
Mean fracture loads (N)	941.80 (±221.66)	534.00 (±110.84)	696.20 (±222.20)
Flexural strength (MPa)	236-600	340-400	—

**Table 4:** Comparison between the properties of some aluminum oxide and zirconium oxide products [48, 74–76].

	Alumina		Zirconia	
	Procera™ AllCeram	In-Ceram AL	VITA In-Ceram® YZ	Lava™ Frame Zirconia
Main component	Al_2_O_3_	Al_2_O_3_	5Y-TZP	3Y-TZP
Fracture toughness (MPa·m^1/2^)	3.50-4.90	5.52-5.70	5.90	3.50-4.50
Vickers hardness (GPa)	17.90-18.90	12.65-13.43	12.65-13.43	—
Modulus of elasticity (GPa)	—	—	200-210	200-210
Fracture strength (N)	784.80-1953.50	—	665-2374	
Indications	Single crown	Single-crown and three-unit bridges for anterior teeth	Single-crown and three-unit anterior and posterior bridges	Single crown, multiunit bridges, inlay bridges, and full-zirconia crowns

## Data Availability

All data, figures, and tables in this review paper are labeled with references.
